# Detection and Correlation Analysis of Serum Uric Acid in Patients with Thyroid-Associated Ophthalmopathy

This article has been retracted.

**DOI:** 10.1155/2022/8406834

**Published:** 2022-09-27

**Authors:** Jingbo Zhou, Xu Yu, Yan Lou, Jinjing Bao, Yuequan Xia, Lin Zhu

**Affiliations:** ^1^Department of Endocrinology, Affiliated Hospital of Nanjing University of Chinese Medicine, Nanjing 210029, China; ^2^School of Graduate, Nanjing University of Chinese Medicine, Nanjing 210023, China; ^3^Physical Examination Center, Affiliated Hospital of Nanjing University of Chinese Medicine, Nanjing 210029, China

## Abstract

**Purpose:**

To probe the property of serum uric acid in evaluating the activity of patients with thyroid-associated ophthalmopathy.

**Methods:**

A total of 443 patients with TAO admitted to our hospital from March 2016 to February 2021 were selected for the observation group. Simultaneously, 443 healthy subjects were selected for the control group. The observation group was divided into the active group (*n* = 254) and the inactive group (*n* = 189) according to the clinical activity score (CAS). Besides, the patients were divided into mild group (*n* = 201), moderate severe group (*n* = 133) and extremely severe group (*n* = 109) based on the severity of TAO. Serum uric acid, free triiodothyronine (FT3), free thyroid hormone (FT4), thyrotropin stimulating hormone (TSH) and glycosylated hemoglobin (HbA1c) levels were detected and analyzed in each group.

**Results:**

Serum UA, FT3, FT4, TSH and HbA1c in the active group were significantly enhanced than those in the other two groups (*P* < 0.05), and there was no significant difference between the inactive group and the control group (*P* > 0.05). In different disease severity groups, the serum UA level of patients in the active group was significantly promoted than that in the inactive group and control group (*P* < 0.05) and was decreased successively in extremely severe group, moderate severe group and mild group, with statistical significance (*P* < 0.05). Pearson's analysis showed that UA was positively correlated with FT3, FT4, and HbA1c (*r* = 0.652, *P* = 0.031; *r* = 0.571, *P* = 0.042; *r* = 0.737, *P* = 0.024), while was reversely correlated with TSH level (*r* = −0.137, *P* = 0.262). There was no correlation between UA and FT3, FT4, and HbA1c levels in the inactive group. UA detection showed the average sensitivity and specificity of TAO activity were 94.3% and 85.2%, respectively. There was no significant correlation between the severity of disease and serum UA in inactive patients (*P* = 0.135). There was a positive correlation between the severity of disease and serum UA in active patients (*P* = 0.005).

**Conclusion:**

UA may be used as a laboratory indicator for quantitative clinical diagnosis of thyroid-associated ophthalmopathy (TAO) and as a parameter for the presence of TAO activity.

## 1. Introduction

Thyroid-associated ophthalmopathy (TAO) belongs to one of the most common orbital diseases, with the highest morbidity in adults. It is generally considered to be an organ-specific autoimmune disease associated with thyroid dysfunction [1]. Its clinical manifestations are mainly eyeball protrusion, contracture of upper eyelid, diplopia, strabismus, optic nerve damage, and so on [2]. The course of TAO is divided into two stages: active phase and quiescent phase [3]. Due to the fact that different treatment methods need to be adopted at different stages of the disease, it is of great significance to evaluate the activity of eye disease for the selection of treatment methods and estimation of prognosis. At present, the evaluation of TAO activity is mainly based on the symptoms and signs of patients, as well as imaging examination, which is easily affected by subjective factors such as patients themselves and ophthalmologists' work experience [4]. Recently, the study of laboratory parameters on TAO activity has made some progress, and it has been reported that urinary glycosaminoglycan (uGAG) and serum uric acid (sUA) play important roles in the evaluation of TAO activity [5, 6]. UA is the final product of the purine metabolism in the human body [7]. sUA levels indicate the balance between the metabolic breakdown of purine nucleotides and UA excretion [8]. sUA levels are considered an independent predictor for metabolic syndrome [9]. However, diverse reports have different conclusions, and the examination method is time-consuming, making it difficult to be routinely applied.

In this study, 443 patients with TAO treated in our hospital were carried on detecting the content of sUA, for the sake of exploring the role of sUA in the evaluation of activity of TAO patients.

## 2. Clinical Data and Methods

### 2.1. General Clinical Data

A total of 443 patients including 233 males and 210 females with TAO admitted to our hospital from March 2016 to February 2021 were selected as the observation group, and 443 healthy people including 225 males and 218 females were chosen as the control group during the same period. All patients obtained informed consent, and the research was reviewed and approved by the medical ethics committee of hospital. The following are the inclusion criteria: (1) The diagnostic criteria of TAO were met. (2) Informed consent was signed by both patients and their families and approved by the hospital's medical ethics committee. (3) There are no conscious disorders and mental disorders. (4) Thyroid function in all patients was within normal range. (5) The intraocular pressure of patients was within a normal range. The following are the exclusion criteria: (1) The presence of internal diseases affecting SUA levels, such as primary gout, malignant tumor, kidney disease, diabetes, and blood diseases; (2) age < 20 or >75 years old; (3) having autoimmune thyroiditis and secondary hyperthyroidism; and (4) pregnant and lactating women.

### 2.2. Methods

#### 2.2.1. Blood Sample Collection

All subjects fasted for 12 h before blood collection, strictly controlled their diet for 1 week before blood collection, and did not eat food with great influence on blood lipid and uric acid. All subjects were collected 5 mL fasting venous blood in the morning after enrollment. Among them, patients in the observation group were added with methylimidazole or propylthiouracil, and their blood was collected again after thyroid function was normal. The blood samples were centrifuged at 3000 r/min for 10 min with an effective centrifugation radius of 6 cm. The serum was routinely separated and stored in a 20°C refrigerator for testing.

#### 2.2.2. Measurements of Blood Glucose and Blood Lipid Levels

Fasting blood glucose (FBG), total cholesterol (TC), triglyceride (TG), high-density lipoprotein cholesterol (HDL-C), and low-density lipoprotein cholesterol (LDL-C) were assessed by the Hitachi 7600 automatic biochemical analyzer.

#### 2.2.3. Determination of Thyroid Hormone and Blood Uric Acid Levels

Levels of serum free triiodothyronine (FT3), free thyroxine (FT4), thyrotropin stimulating hormone (TSH), and glycosylated hemoglobin (HbA1c) in both groups were detected by electrochemiluminescence immunoassay (Roche, Cobas E601). The serum uric acid levels of the two groups were determined by uric acid oxidase-peroxidase method.

#### 2.2.4. TAO Subgroups

Patients in the observation group were divided into two groups according to the difference in clinical activity score (CAS) [10]. If CAS score reached 4, patients were selected in the active stage; otherwise, patients were in the inactive stage. Among which, 254 cases were in the active stage and 189 cases were in the inactive stage. Meanwhile, the patients were divided into the mild group (*n* = 201), the moderate severe group (*n* = 133), and the extremely severe group (*n* = 109) according to the severity of TAO. TAO has three levels of severity: mild, moderate-severe, and very severe (threatening vision). Based on one or more of the following: mild or sufficient interference with daily life, eyelid pullback ≥ 2 mm, soft tissue involvement, higher than normal, unstable or persistent diplopia ≥ 3 mm, corneal contact lubricant reaction, thyroid dysfunction optic neuropathy, and/or corneal rupture. After statistical analysis, there was no significant difference in age, gender and other general clinical data of each group, which was comparable.

### 2.3. Statistical Analysis

SPSS21.0 was used for data analysis. The assessment data of FBG, TC, TG, HDIL-C, LDL-C, FT3, FT4, TSH, and blood uric acid levels in the two groups were in line with normal distribution by a normality test and were described by *Z* ± *S*. A group *t*-test was used for intergroup comparison, and a paired *t*-test was used for intragroup comparison. Correlation was analyzed by Pearson's correlation analysis. The test standard *α* = 0.05; *P* < 0.05 was statistically significant.

## 3. Results

### 3.1. Comparison of UA, FT3, FT4, TSH, and HbA1c between the CAS Group and Control Group

As indicated in Figure 1, serum UA, FT3, FT4, TSH, and HbA1c in the active group were significantly elevated than those in the other two groups (*P* < 0.05), and there was no statistical significance between the inactive group and the control group (*P* > 0.05).

### 3.2. Comparison of UA Levels between Patients with Different Degree of Disease and CAS Stage and Control Group

As revealed in Table 1, in the groups of different severity of disease, serum UA level in the active patients was significantly promoted than that in the inactive patients and the control group (*P* < 0.05), and was decreased successively in the extremely severe group, the moderate severe group and the mild group, with statistical significance (*P* < 0.05).

### 3.3. Correlation between UA and FT3, FT4, TSH, and HbA1c in the CAS Group

As unveiled in Figure 2, Pearson's analysis uncovered that UA was positively correlated with FT3, FT4, and HbA1c (*r* = 0.652, *P* = 0.031; *r* = 0.571, *P* = 0.042; *r* = 0.737, *P* = 0.024), whereas was inversely correlated with TSH level (*r* = −0.137, *P* = 0.262). UA in the inactive group had no correlation with FT3, FT4, and HbA1c levels.

### 3.4. OC Curve Analysis of UA in TAO Patients

As shown in Figure 3, the area of UA under ROC curve in TAO patients was 0.941. The average sensitivity and specificity of UA were 94.3% and 85.2%, respectively. The activity of 443 patients with TAO matched the diagnosis of 402 cases.

### 3.5. Correlation Analysis between the Disease Severity of Active Period and UA

As demonstrated in Table 2, there was no significant correlation between the severity of disease and serum UA in inactive patients (*P* = 0.135). There was a positive correlation between the severity of disease and serum UA in active patients (*P* = 0.005).

## 4. Discussion

TAO is an autoimmune disease of which thyroid and orbital tissues produce common antigens leading to T cells and cytokine-mediated autoimmune reactions, characterized by infiltration of lymphocytes and plasma cells, stimulation of proliferation of orbital fibroblasts, and secretion of GAG accumulation in orbit, that is, secretory deposition and tissue edema (inflammatory active phase), and in the later stage, fibrogenesis (quiescent phase). Due to the accumulation of a large number of hydrophilic macromolecular substances, aminoglucosan results in extraocular muscle edema, thereby increasing the pressure behind the eye, and results in the eyeball protrusion of patients. Moreover, limited extraocular muscle activity due to edema causes a series of symptoms, such as diplopia, extraocular muscle contracture, corneal exposure, and eye movement disorders with eyelids unable to close [11–13].

TAO is a wasting disease. Patients in the active stage are in a high metabolic state for a long time and consume more adenosine triphosphate (ATP) than normal people, leading to the increased production of uric acid. It can be seen from the pathway of purine metabolism that ATP participates in the process of uric acid metabolism. ATP metabolism will form ADP or AMP. Under normal conditions, the rates of AMP synthesis and decomposition are similar, so that the daily uric acid production is constant. If the body occurs hypermetabolic states such as hyperthyroidism, ATP will be consumed in large quantities, resulting in the production of AMP and increased production of uric acid, thus causing inflammation in the body. As reported previously, the ocular deposition of GAG in TAO patients is mainly HA [14]. TAO patients not only have glycosaminoglycan deposition in orbital tissues but also have increased blood and uric acid levels. Therefore, serum UA was selected as the measurement index in this study. Recently, UA is closely associated with thyroid dysfunction [15]. In a recent cross-sectional study, UA has a positive correlation with thyroid nodules [16]. Moreover, various studies have found that the change of serum uric acid level is related to the incidence and mortality of diabetes, cardiovascular diseases, renal diseases, and various clinical syndromes [17, 18]. Hyperuricemia is also an important component of metabolic syndrome [19, 20]. It has been reported that sUA in the TAO group is higher than that in healthy age- and sex-matched volunteers [21]. Consistently, the results in this research unmasked that the concentration of UA in the active TAO group was significantly enhanced than that in the static TAO group and the normal control group (*P* < 0.05), which was 2.38 times of that in the static TAO group and 2.80 times of that in the normal control group. Furthermore, there was no significant difference of serum UA concentration between the static TAO group and the normal control group (*P* > 0.05), which was in line with the existing research views [22, 23]. This indicated that patients in the active TAO group had inflammation in eyelid and thyroid, and UA production rate could be increased. However, serum UA expression of patients in the inactive TAO group was normal, which may be related to the fade of inflammatory cell infiltration during this period. This study also proved that in the groups of different severity of disease, serum UA level in the active patients was significantly increased than that in the control group and was decreased successively in the extremely severe group, the moderate severe group, and the mild group (*P* < 0.05). These results mirrored that the more severe condition of active TAO patients, the higher the serum UA expression level was. For active TAO patients, the degree of illness can affect the expression of UA. In this paper, correlation analysis suggested that there was a significant positive correlation between the severity of disease and serum UA expression in active patients (*P* = 0.005). As we know, FT3, FT4, and HbA1c are important indexes for assessing thyroid function [24]. In our study, we found that UA in active patients was positively correlated with FT3, FT4, and HbA1c (*r* = 0.652, *P* = 0.031; *r* = 0.571, *P* = 0.042; *r* = 0.737, *P* = 0.024), while it was negatively correlated with TSH level (*r* = −0.137, *P* = 0.262). However, inactive patients had no such correlation (*P* = 0.135), and UA in the inactive group had no correlation with FT3, FT4, and HbA1c levels (*P* > 0.05), which was consistent with existing research views. This indicated that the UA level was increased with the aggravation of disease during active TAO period.

The two most basic indicators of diagnostic value are sensitivity and specificity. ROC curve can evaluate the efficiency of a test from these two aspects and directly reflect the area under the curve, which is convenient for comparison between different methods. The area under ROC curve is used to evaluate the accuracy of the diagnostic experiment. According to Swets criteria, the area below 0.5 indicates that the experiment has no diagnostic value, the area between 0.5 and 0.7 has a low accuracy, the area between 0.7 and 0.9 has a certain accuracy, and the area > 0.9 has a high accuracy. This paper showed that the area of UA under the ROC curve was 0.941, suggesting that all UA indicators had high diagnostic value.

This study has some limitations: the sample size of is small, and the current results can only draw preliminary conclusions. In the near future, the sample size should be expanded and the detailed group studies should be conducted to explore the dose-response relationship.

Above all, UA levels of patients in active TAO stage was obviously enhanced than that of motionless phase and the normal control group, and the difference was statistically significant, which showed that UA was involved in the pathological process of TAO patients. Besides, the serum UA level in TAO group was promoted with the increase of the severity of eye disease, which indicated that both of them were closely correlated with the incidence of TAO and were positively correlated with the severity of secretory ophthalmopathy. Our study suggested that UA could be used as a laboratory index for clinical diagnosis of TAO patients and a parameter for the activity of TAO and provided a basis for exploring the value of UA level and its changes in the clinical therapeutic effect and prognosis evaluation of TAO.

## Figures and Tables

**Figure 1:** Comparison of UA, FT3, FT4, TSH, and HbA1c between the CAS group and control group.

**Figure 2:** Correlation between UA and FT3, FT4, TSH, and HbA1c in CAS group.

**Figure 3:** OC curve analysis of UA in TAO patients.

**Table 1:** Comparison of UA levels between CAS stage patients with different disease severity and control group.

Groups	n	Inactive period	Active period
Control group	443	271.82 ± 60.45	
Mild group	201	279.46 ± 62.67	294.33 ± 65.33
Moderate severity group	133	302.21 ± 72.44	325.43 ± 71.55
Severity group	109	327.59 ± 68.48	372.25 ± 63.45

**Table 2:** Correlation analysis between the disease severity of active period and UA.

Project	UA	
	*r*	*P*
Inactive patient severity	0.102	0.135
Active patient severity	0.695	0.005

## Data Availability

Original data included/analyzed in this study are available from the corresponding author under reasonable requests.
